# Adrenal Gland Infection by Serotype 5 Adenovirus Requires Coagulation Factors

**DOI:** 10.1371/journal.pone.0062191

**Published:** 2013-04-25

**Authors:** Lucile Tran, Laure-Hélène Ouisse, Peggy Richard-Fiardo, Philippe R. Franken, Jacques Darcourt, Gaétan Cornilleau, Karim Benihoud, Georges Vassaux

**Affiliations:** 1 INSERM U948, Nantes, France; 2 Faculté de Médecine, Université de Nice-Sophia-Antipolis, Nice, France; 3 UMRE4320, CEA, Nice, France; 4 Université Paris-Sud, UMR 8203, Institut Gustave Roussy, Villejuif Cedex, France; Justus-Liebig-University Giessen, Germany

## Abstract

Recombinant, replication-deficient serotype 5 adenovirus infects the liver upon *in vivo*, systemic injection in rodents. This infection requires the binding of factor X to the capsid of this adenovirus. Another organ, the adrenal gland is also infected upon systemic administration of Ad, however, whether this infection is dependent on the cocksackie adenovirus receptor (CAR) or depends on the binding of factor X to the viral capsid remained to be determined. In the present work, we have used a pharmacological agent (warfarin) as well as recombinant adenoviruses lacking the binding site of Factor X to elucidate this mechanism in mice. We demonstrate that, as observed in the liver, adenovirus infection of the adrenal glands *in vivo* requires Factor X. Considering that the level of transduction of the adrenal glands is well-below that of the liver and that capsid-modified adenoviruses are unlikely to selectively infect the adrenal glands, we have used single-photon emission computed tomography (SPECT) imaging of gene expression to determine whether local virus administration (direct injection in the kidney) could increase gene transfer to the adrenal glands. We demonstrate that direct injection of the virus in the kidney increases gene transfer in the adrenal gland but liver transduction remains important. These observations strongly suggest that serotype 5 adenovirus uses a similar mechanism to infect liver and adrenal gland and that selective transgene expression in the latter is more likely to be achieved through transcriptional targeting.

## Introduction

Recombinant, serotype 5 adenoviruses are probably the most widely used delivery vectors in gene therapy. *In vitro* and *in vivo* upon local injection, they can infect a wide range of cell types such as epithelial cells [1], [2], [3], cardiomyocytes [4] and cancer cells [5], [6], [7], [8]. *In vivo*, systemic injection of recombinant adenovirus is followed by a rapid disappearance of the virus from the blood stream [9] and leads to a predominant expression in hepatocytes [10], [11], [12], [13], [14]. Another organ efficiently infected by adenoviruses upon systemic injections is the adrenal glands [15], [16], [17], [18], [19]. Although the infectivity of the adrenal gland is below that of the liver [18], it is equivalent to that of the spleen [17]. In the adrenal gland, the site of synthesis of cortisol and corticosterone, the *zona fasciculata,* has been shown to be particularly prone to infection [18].

Classically, the sequence of *in vitro* infection of an adenovirus serotype 5 is thought to involve the binding of the viral fiber to the coxsackie adenovirus receptor (CAR), followed by internalization mediated by cellular αv-integrins [20], [21]. If the sequence of events involved for *in vivo* infection was initially thought to be similar to the *in vitro* one, recent data have changed the overall consensus: Despite a strong expression of CAR in the liver [22], conflicting results using capsid-modified adenoviruses were reported [10], [23], [24] questioning the role of CAR in adenovirus infection of the liver *in vivo*. Since then, different studies have demonstrated a role of vitamin K-dependent blood factors in liver transduction [25], [26], [27], [28], [29]. More precisely, this phenomenon was attributed to factor X (FX) binding to capsid hexon protein, making a bridge between the virus and hepatocyte heparan sulfate glycosaminoglycans [25], [26], [27], [28], [29].

Although adrenal glands can be infected through systemic administration of the virus, the level of transgene expression achieved remains low. This modest level of transgene expression is illustrated by the fact that gene transfer in the adrenal glands cannot be visualized by sensitive, whole-body imaging techniques such as PET or even SPECT using the Na/I symporter (NIS) as a reporter gene, while transgene expression in the liver can easily be detected and quantified using either of these methodologies [30], [31]. Two strategies could be envisaged to restrict and/or increase transgene expression in the adrenal gland: i) selective transduction of the adrenal glands, but, for this strategy to be efficient, the mechanism of infection of the two organs would have to be different and ii) a more localized type of injection (i.e. direct injection in the kidney) would increase the viral load in the vicinity of the adrenal gland and potentially increase transduction.

In this context, the aim of the present study is to gain a better understanding of the transduction of the adrenal glands by type 5 adenovirus and to assess a new administration routes to improve adrenal gland transduction by this vector.

## Materials and Methods

### Adenovirus

The replication-incompetent adenovirus, Ad-CMV-rNIS, in which the immediate-early promoter of CMV drives the expression of rat NIS, has been described previously [32]. Ad-CMV-nls-LacZ, is a recombinant, replication deficient adenovirus in which the expression of the β-galactosidase gene containing a nuclear localization signal is driven by the immediate-early CMV promoter. Both viruses were produced and titrated at the “Plateforme de production de vecteurs pré-cliniques du CHU de Nantes”, using a standard protocol.

### Animals Studies

Animal housing and procedures were conducted according to the guidelines of the French Agriculture Ministry and were approved by the institutional review board (CIEPAL: Comité Institutionnel d’Ethique Pour l’Animal de Laboratoire) (Permit number # A06-088-14). Gene-transfer studies were performed on female Balb/c mice obtained at 8 weeks of age from Janvier (Le Genest Saint Isle, France). Ad-CMV-rNIS (5×10^8^ or 1×10^9^ PFU/mouse) in sterile saline buffer (final volume, 200 µl) was administered intravenously. For the intra-renal injections, Ad-CMV-rNIS (5×10^8^ PFU/mouse) were injected into the parenchyma of the left kidney of anaesthetised, 7-week-old Balb/c mice. For biodistribution studies, mice were also injected subcutaneously (s.c.) with 133 µg of warfarin/mouse 3 and 1 day prior to Ad vector injections as previously described [25].

### MicroSPECT/CT Studies

Forty eight hours after adenovirus administration, mice were injected intraperitoneally with 100 MBq ^99m^Tc pertechnetate (^99m^TcO_4_^−^) obtained from a freshly eluted ^99^Mo/^99m^Tc generator. Precisely 20 min later, mice were imaged under Isofluran anaesthesia (Baxter, Aerane). Localization of the kidney was performed using ^99m^Tc-Dimercaptosuccinic acid (^99m^Tc-DMSA) as a probe. Briefly, DMSA (TechneScan DMAS) was labelled using a standard procedure [33]. This tracer (95 MBq) was administered by intraperitoneal injection. Five hours later, the animals were anaesthetized and scanned. In both cases (^99m^Tc pertechnetate and ^99m^Tc-DMSA) SPECT/CT scans were performed using a micro-SPECT-CT (eXplore speCZT CT120, General Electric), using a previously published protocol [31]. Image analyses and quantification were performed using the ‘AMIDE’ software [34].

### Enzymatic and PCR Assays

β-galactosidase activity was measured as previously described [29]. Total RNA from the livers or adrenal glands of adenovirus-injected mice were extracted using Nucleospin RNAII (Macherey-Nagel, France) and transcribed into cDNA using the Superscript III enzyme (Invitrogen, France). CAR and 18S expression were determined using primers and experimental conditions described in [35] and [36], respectively. Real-time PCR was performed with the 7900HT Fast Real-Time PCR System and carried out using TaqMan® gene expression assays (Applied Biosystem, France). Primer sets (Rn 00583900-m1 for NIS and Mm-013518-11 for GAPDH) were designed by, and purchased from, Applied Biosystems. Cycle parameters were 95°C for 20 s followed by 40 cycles of 95°C for 1 s and 60°C for 20 s. Relative mRNA expression levels were determined using ΔCt values obtained by subtracting Ct control (mouse GAPDH) from Ct target gene (rat NIS), measured in the same RNA preparation.

## Results

### Adenovirus Infection of the Adrenal Gland is CAR-independent

We first assessed whether the CAR receptor is expressed in the adrenal glands. For that purpose, mRNA was extracted from dissected adrenal glands or a liver biopsy (as a positive control) and subjected to reverse-transcription and PCR amplification. As expected, CAR is indeed expressed in the liver (Figure 1A). By contrast, in the adrenal glands, CAR is undetectable (Figure 1A).

**Figure 1:** A: CAR expression in the liver and the adrenal glands. Total RNAs were extracted from liver biopsies or total adrenal glands and subjected to reverse transcription and PCR amplification. The PCR products were separated by electrophoresis. B and C: Mice were injected systemically with 10^9^ PFU of either AdHwt (n = 7) or AdH[GA]24 (n = 7) or PBS (n = 4). Forty-eight hours later, the animals were culled and the livers and adrenal glands were collected. B: Whole liver were stained for β-galactosidase expression. C: Total RNA were extracted from the adrenal glands (two glands from the same animal were pooled), reversed-transcribed and subjected to quantitative PCR to detect LacZ expression or 18S RNA. The ratio LacZ/18S of adrenal glands collected from animals injected with AdHwt was used as 100%. The data presented are means+SEM. Statistical test: ANOVA (Prism, Graph-Pad softwares).

To exclude completely a CAR-dependent mechanism and provide new insight into the infection of the adrenal glands, we compared transgene expression upon injection of a wild-type, replication-deficient adenovirus (AdHwt, 10^9^ PFU) and a replication-deficient adenovirus in which the hexon hypervariable region 5 had been modified (AdH[GA]24, 10^9^ PFU). Both viruses encode the LacZ gene driven by the same promoter and both are equally able to infect CAR-positive cells [29]. β-galactosidase staining of the whole liver obtained forty-eight hours after systemic AdHwt injection showed an intense blue colour, characteristic of LacZ gene expression (Fig. 1B), while staining of a liver obtained from an AdH[GA]24-injected animal remained unstained (Fig. 1B). This set of results confirms previous data by Vigant et al [29] and highlights the requirement of functional hexon proteins for adenovirus infection, *in vivo*. In the adrenal glands, systemic administration of AdHwt resulted in a very significant increase in β-galactosidase expression compared to untreated controls, while systemic injection of AdH[GA]24 resulted in levels of β-galactosidase transcripts fifty times lower than those obtained with AdHwt (Fig. 1C; P<0.001). Altogether, these results demonstrate that, in contrast to the wild-type AdHwt, AdH[GA]24 is unable to transduce either the liver (Fig. 1B) or the adrenal glands (Fig. 1C). These data strongly suggest that, as in the liver, infection of the adrenal glands involves blood factors that bind to the viral capsid.

### Involvement of Blood Factors in Adenovirus Infection of the Adrenal Glands

To determine whether blood factors are indeed involved in the infection of the adrenal glands by type 5 adenovirus, a pharmacological intervention (warfarin pre-treatment) was used. Warfarin inhibits the vitamin K-dependent γ carboxylation of the glutamic acid residues in the N-termini of Factor II, VII, IX and X as well as protein C and results in reduced functional, circulating levels of these coagulation factors. To compare the effect of warfarin on adenovirus-mediated gene transfer in the liver and the adrenal glands, warfarin was administered three and one days before virus administration. Twenty-four hours after the last injection of warfarin, the animals were administered intravenously with 6×10^8^ PFU of Ad-CMV-nls-LacZ. As expected, systemic injection of this virus led to strong levels of β-galactosidase activity in the liver (Figure 2A). Pre-treatment of the experimental animals with warfarin reduced dramatically this activity (Figure 2A). In the adrenal glands, systemic administration of Ad-CMV-nls-LacZ resulted in a significant increase in β-galactosidase activity that was significantly reduced (p<0.05) by warfarin pre-treatment (Figure 2A). RT-qPCR to measure β-galactosidase transcripts levels on mRNA extracted from the liver or the adrenal glands of warfarin-treated or non-treated animals confirmed these data (Figure 2B). In both cases, warfarin pre-treatment reduced β-galactosidase-specific mRNA expression by more than a factor 10 (Figure 2B). These results suggest that blood factors are required not only for efficient transduction of liver but also for adrenal glands transduction by adenovirus type 5.

**Figure 2:** **Effect of warfarin pre-treatment on adenoviral transgene expression.** A replication-deficient recombinant adenovirus encoding the Lac-Z gene (6×10^8^ PFU) was injected in control- (Adenovirus) or warfarin-pretreated animals (Warfarin and Adenovirus). Twenty-four hours later, liver biopsies or adrenal glands were collected. A: Measurement of the β-galactosidase protein in the samples was performed. The data presented are percentages of mean +/− SEM from untreated animals (n = 2), adenovirus-injected animals (n = 10) and adenovirus-injected animals, pre-treated with warfarin (n = 10). 100% represents the average of β-galactosidase activity in the adrenal glands (100% = 7584 β-gal units/mg of protein) or liver (100% = 24805 β-gal units/mg of protein) of adenovirus-injected animals. Statistical test: ANOVA (Prism, Graph-Pad softwares). B) Total RNA were collected from individual adrenal glands or liver biopsies, reversed-transcribed and subjected to quantitative PCR to detect LacZ or 18S RNA. The ratio LacZ/18S of liver or adrenal glands collected from animals injected with adenovirus was set at 100%. Data presented are duplicate determinations from a single adrenal gland and liver biopsy and is representative of 4 independent experiments.

### Involvement of Factor X

To determine whether factor X can restore gene transfer abolished by warfarin, 6×10^8^ PFU of Ad-CMV-nls-LacZ were injected systemically in warfarin-treated mice or warfarin-treated mice supplemented with 33 µg of recombinant factor X (Haematologic Technologies, Essex Junction, VT, USA) (intravenous injection) prior to adenovirus administration. Forty-eight hours later, experimental animals were culled and livers and adrenal glands were collected. Figure 3A shows that factor X administration restores the transduction of the liver, measured by β-galactosidase staining of the whole organ. The same phenomenon can be observed in the adrenal gland of these animals, as the levels of LacZ transcripts are nearly ten times higher in the adrenal glands of factor X-complemented animals than in the adrenal glands of warfarin control animals (Fig. 3B). These results demonstrate that the mechanism of infection of the adrenal glands by adenovirus requires, as observed for the liver, a complex between factor X and the viral particle.

**Figure 3:** Influence of Factor X on adenovirus transduction in warfarin-treated mice. A replication-deficient recombinant adenovirus encoding the Lac-Z gene (6×10^8^ PFU) was injected in warfarin-pretreated animals (n = 7) or warfarin-pre-treated, factor X-complemented animals (n = 5). Forty-eight hours later, liver biopsies or adrenal glands were collected. A) Whole liver were stained for β-galactosidase expression. B: Total RNA were extracted from the adrenal glands (two glands from the same animal were pooled), reversed-transcribed and subjected to quantitative PCR to detect LacZ expression or 18S RNA. The ratio LacZ/18S of adrenal glands collected from warfarin-pre-treated, factor X-complemented animals injected with adenovirus was set at 100%. The data presented are means+SEM. Statistical analysis: Student t test (Prism, Graph-Pad softwares).

### Visualization of the Kidneys by SPECT/CT

The SPECT tracer ^99m^Tc-dimercaptosuccinic acid (^99m^Tc-DMSA) is used in nuclear medicine to visualize the renal cortex [33]. This tracer was injected to mice. Five hours later, the animals were anaesthetized and subjected to a SPECT/CT scan. Figure 4A show transverse, coronal and sagittal views of the accumulation of ^99m^Tc-DMSA in the kidneys. A three-dimensional reconstruction of the images is also presented (Figure 4B). Altogether, the information obtained allow a localization of the kidneys in the SPECT/CT images which can in turn be use for an accurate localization of the adrenal glands.

**Figure 4:** Localization of the kidneys using ^99m^Tc-DMSA. Mice were injected intra-peritoneally with 95 MBq of ^99m^Tc-DMSA. Five hours later, the animals were anaesthetized and SPECT/CT scans performed. A) Transverse, coronal and sagittal sections centered on the kidneys. B) Volume rendering of the whole animal in which the kidneys appear in yellow. Legend: K: kidney, L: left, post: posterior side of the animal.

### Adrenal Glands Transduction Upon Intra-renal Injection of Adenovirus Type 5 is Detectable by SPECT/CT Imaging and is Warfarin-dependent

To investigate whether intra-renal administration of adenovirus could lead to improved transduction, mice were injected with 5×10^8^ PFU of Ad-CMV-rNIS in the left kidney. Forty-eight hours later, the animals were administered intra-peritoneally with the tracer ^99m^TcO_4_^−^. This tracer accumulates selectively in organs expressing the Na/I symporter (NIS) [31], i.e the thyroid, stomach and salivary glands that express NIS endogenously as well as the organs/tissues transduced by the adenovector. The animals were then anaesthetized and positioned into a SPECT/CT scanner.

The SPECT/CT images, analyzed in the light of the images obtained using the kidney specific probe ^99m^Tc-DMSA (Figure 4), revealed a strong, discrete signal just above the kidney, in an area expected to encompass the adrenal gland (Figure 5A). As such a signal is absent in SPECT/CT images of mice administered intravenously with the same adenovirus [31] or in the contra-lateral kidney (not shown), this set of data suggests that the intra-renal route of administration of adenovirus is more efficient than the intravenous one to transduce this organ. A similar imaging protocol involving intra-renal administration of 5×10^8^ PFU of Ad-CMV-rNIS in mice pre-treated with warfarin resulted in a lack of signal in the adrenal glands area (Figure 5B), confirming that adrenal gland infection depends on blood factors. Images focusing on the liver showed that intra-renal administration of Ad-CMV-rNIS led to an important transduction of this organ (Fig. 6A). Quantitative analysis of liver adenoviral transduction in animals administered using the intra-venous or intra-renal route failed to show any statistically-significant difference. In addition, SPECT/CT analysis of the liver of animals administered intra-renal with Ad-CMV-rNIS confirmed that liver transduction is warfarin dependent (Fig. 6B). To verify the data obtained through imaging, analysis of transgene expression was performed using quantitative RT-PCR on liver and adrenal gland biopsies. The data presented in Figure 7 confirm the imaging data and demonstrate that the intra-renal route of administration results in the transduction of the adrenal glands and that both liver and adrenal gland transduction are warfarin-dependent.

**Figure 5:** Visualization of gene transfer in the adrenal gland upon intra-renal injection: Effect of warfarin. Direct injection of 5×10^8^ PFU Ad-CMV-rNIS in the left kidney was performed on control (A) or warfarin-treated mice (B). Forty-eight hours later, the mice were anaesthetized and SPECT/CT scans performed. The transverse, coronal and sagittal sections presented are centered on the adrenal glands. Legend: AG: adrenal glands, L: liver, K: kidneys, S: stomach, post: posterior side of the animal.

**Figure 6:** Visualization of gene transfer in the liver upon intra-renal injection: Effect of warfarin. Direct injection of 5×10^8^ PFU Ad-CMV-rNIS in the left kidney was performed on control (A) or warfarin-treated mice (B). Forty-eight hours later, the mice were anaesthetized and SPECT/CT scans performed. The transverse, coronal and sagittal sections presented are centered on the liver. Legend: L: liver, S: Stomach.

**Figure 7:** Effect of warfarin pre-treatment on adenoviral transgene expression following intra-renal administration. Ad-CMV-rNIS, a replication-deficient recombinant adenovirus encoding the NIS gene (5×10^8^ PFU) was injected into the left kidney of control- (Adenovirus) or warfarin-pretreated animals (Warfarin and Adenovirus). Fourty-eight hours later, liver biopsies and adrenal glands were collected. Total RNA were collected from individual adrenal glands (on the left kidney) or liver biopsies, reversed-transcribed and subjected to quantitative PCR to detect rNIS expression or GAPDH RNA. The ratio rNIS/GAPDH of liver or adrenal glands collected from animals injected with adenovirus was set at 100%. Data presented are triplicate determinations from three adrenal gland and liver biopsies. The data presented are means+SEM. Statistical analysis: Student t test (Prizm, Graph-Pad softwares). **p≤0,01.

## Discussion

Although adenovirus infection has been thought, for more than a decade, to require the binding of the virus to the cellular CAR, recent data have demonstrated that, *in vivo*, when the virus is administered systemically, CAR is not required for infection. The current consensus describes the formation of a complex between the adenovirus and a blood factor (factor X) and this complex is taken up by cells in a CAR-independent mechanism. This concept has been elucidated in the liver but has also been demonstrated in the spleen [26], lung and heart [37], [38] and human epithelial cells [39] and involves heparan sulfate proteoglycans [40]. In the adrenal glands, CAR mRNA is undetectable (Figure 1A). This result is in agreement with previous work describing the lack of CAR-specific immuno-reactivity in mouse adrenal glands [41] and suggests strongly that the infection of the adrenal glands by adenovirus type 5 is CAR-independent. Subsequent experiments using both capsid-modified adenoviruses and pharmacologic interventions confirmed this hypothesis and demonstrated that adenovirus infection in this tissue depends on Factor X. Therefore, our data demonstrate that the adrenal glands are infected in a way similar to that described for infection of the liver, spleen, lung, heart and human epithelial cells. In this context, our data strengthen the point of view suggesting the general nature of this mechanism.

To our knowledge, this is the first time that the warfarin-sensitive nature of adenovirus infection *in vivo* as well as transduction of the adrenal glands by any gene delivery vector was demonstrated using imaging of gene expression. In this context, monitoring of gene transfer using NIS as a reporter gene by SPECT/CT offers many advantage. This methodology allows repetitive, longitudinal studies of transgene expression [31] and has also been used and validated to monitor the spread of oncolytic virus [7], [42]. Humans and clinical trials have validated the utilization of the NIS reporter gene to monitor cancer gene therapy [43] and to adjust treatment [44]. The data presented in the present work demonstrates that the detection of NIS expression can benefit from the utilization of well-established SPECT probes in nuclear medicine such as ^99m^Tc-DMSA to help to locate transgene expression.

Local delivery of adenovector, through intra-renal injection, results in an increased transduction of the adrenal gland. SPECT/CT imaging of gene expression using this route to administer a replication-deficient adenovirus encoding the Na/I symporter led to a clear, discrete signal in the kidney area. The transduction of the adrenal glands was verified by RT-PCR on biopsies and RT-PCR on mRNAs extracted from the kidneys failed to provide any signal. Quantitative analysis of the images suggested that transgene expression was increased by a factor varying from two to five with the intra-renal route of administration. Considering the short half-life of adenoviruses in the circulation [9], the difference of transduction observed with the two modes of injection is likely to be due to the increased availability of the vector in the adrenal glands. More specifically, upon intra-renal administration, the adenovector probably ends up in the circulation and that the first “transduceable” organ that it encounters is the adrenal glands, followed by the liver. Consistent with this hypothesis and considering the dramatic difference in size of the liver versus the adrenal glands, it is not surprising that the intra-renal or intra-venous mode of administration led to a level of transduction that was not statistically different (not shown). Therefore, the intra-renal route is relevant to increase adrenal gland transduction but is inefficient at reducing liver transduction.

Adenoviral infection of the adrenal glands has been exploited in pre-clinical gene therapy protocols for diseases related to adrenal dysfunctions [45], [46]. Alternatively, infection of the adrenal glands can also be seen as a source of side-effect of an adenoviral gene therapy approach targeting another organ: Adenoviral infection of cells from the adrenal glands has been shown to induce inflammatory cytokines [47], as well as affecting steroid hormone production [47], [48]. In the latter context, the availability of an adenovector that would avoid selectively the transduction of the adrenal glands would prevent potential undesired effects. Reciprocally, an adenovector capable of selective transduction of the adrenal glands would be a useful tool. However, considering that the mechanism of infection appears to be the identical in all tissues infectable in vivo, the best strategy to restrict transgene expression to the adrenal glands is transcriptional targeting rather that targeted transduction. For this purpose, liver-specific [49] or adrenal specific [50] promoter fragments have already been described and may be envisaged.

## References

[1] CohenCJ, ShiehJT, PicklesRJ, OkegawaT, HsiehJT, et al (2001) The coxsackievirus and adenovirus receptor is a transmembrane component of the tight junction. Proc Natl Acad Sci U S A 98: 15191–15196.1173462810.1073/pnas.261452898PMC65005

[2] MerronA, PeerlinckI, Martin-DuqueP, BurnetJ, QuintanillaM, et al (2007) SPECT/CT imaging of oncolytic adenovirus propagation in tumours in vivo using the Na/I symporter as a reporter gene. Gene Ther 14: 1731–1738.1796016110.1038/sj.gt.3303043

[3] WaltersRW, FreimuthP, MoningerTO, GanskeI, ZabnerJ, et al (2002) Adenovirus fiber disrupts CAR-mediated intercellular adhesion allowing virus escape. Cell 110: 789–799.1229705110.1016/s0092-8674(02)00912-1

[4] LiL, OkadaH, TakemuraG, KosaiK, KanamoriH, et al (2009) Postinfarction gene therapy with adenoviral vector expressing decorin mitigates cardiac remodeling and dysfunction. Am J Physiol Heart Circ Physiol 297: H1504–1513.1968418910.1152/ajpheart.00194.2009

[5] WangY, ThorneS, HannockJ, FrancisJ, AuT, et al (2005) A novel assay to assess primary human cancer infectibility by replication-selective oncolytic adenoviruses. Clin Cancer Res 11: 351–360.15671566

[6] PeerlinckI, Amini-NikS, PhillipsRK, IggoR, LemoineNR, et al (2008) Therapeutic potential of replication-selective oncolytic adenoviruses on cells from familial and sporadic desmoid tumors. Clin Cancer Res 14: 6187–6192.1882949710.1158/1078-0432.CCR-08-0410PMC2575844

[7] MerronA, BarilP, Martin-DuqueP, de la ViejaA, TranL, et al (2010) Assessment of the Na/I symporter as a reporter gene to visualize oncolytic adenovirus propagation in peritoneal tumours. Eur J Nucl Med Mol Imaging 37: 1377–1385.2014061210.1007/s00259-009-1379-3

[8] MartinicoSC, JezzardS, SturtNJ, MichilsG, TejparS, et al (2006) Assessment of endostatin gene therapy for familial adenomatous polyposis-related desmoid tumors. Cancer Res 66: 8233–8240.1691220310.1158/0008-5472.CAN-06-1209

[9] AlemanyR, SuzukiK, CurielDT (2000) Blood clearance rates of adenovirus type 5 in mice. J Gen Virol 81: 2605–2609.1103837010.1099/0022-1317-81-11-2605

[10] AlemanyR, CurielDT (2001) CAR-binding ablation does not change biodistribution and toxicity of adenoviral vectors. Gene Ther 8: 1347–1353.1157157210.1038/sj.gt.3301515

[11] Groot-WassinkT, AboagyeEO, WangY, LemoineNR, KeithWN, et al (2004) Noninvasive imaging of the transcriptional activities of human telomerase promoter fragments in mice. Cancer Res 64: 4906–4911.1525646210.1158/0008-5472.CAN-04-0426

[12] PeerlinckI, MerronA, BarilP, ConchonS, Martin-DuqueP, et al (2009) Targeted radionuclide therapy using a Wnt-targeted replicating adenovirus encoding the Na/I symporter. Clin Cancer Res 15: 6595–6601.1986146510.1158/1078-0432.CCR-09-0262

[13] CoughlanL, VallathS, SahaA, FlakM, McNeishIA, et al (2009) In vivo retargeting of adenovirus type 5 to alphavbeta6 integrin results in reduced hepatotoxicity and improved tumor uptake following systemic delivery. J Virol 83: 6416–6428.1936932610.1128/JVI.00445-09PMC2698540

[14] DescampsD, BenihoudK (2009) Two key challenges for effective adenovirus-mediated liver gene therapy: innate immune responses and hepatocyte-specific transduction. Curr Gene Ther 9: 115–127.1935586910.2174/156652309787909544

[15] ChaoJ, ZhangJJ, LinKF, ChaoL (1998) Human kallikrein gene delivery attenuates hypertension, cardiac hypertrophy, and renal injury in Dahl salt-sensitive rats. Hum Gene Ther 9: 21–31.945823910.1089/hum.1998.9.1-21

[16] ThemisM, SchneiderH, KiserudT, CookT, AdebakinS, et al (1999) Successful expression of beta-galactosidase and factor IX transgenes in fetal and neonatal sheep after ultrasound-guided percutaneous adenovirus vector administration into the umbilical vein. Gene Ther 6: 1239–1248.1045543210.1038/sj.gt.3300970

[17] Groot-WassinkT, AboagyeEO, GlaserM, LemoineNR, VassauxG (2002) Adenovirus biodistribution and noninvasive imaging of gene expression in vivo by positron emission tomography using human sodium/iodide symporter as reporter gene. Hum Gene Ther 13: 1723–1735.1239662510.1089/104303402760293565

[18] WangY, Groot-WassinkT, LemoineNR, VassauxG (2003) Cellular characterization of the tropism of recombinant adenovirus for the adrenal glands. Eur J Clin Invest 33: 794–798.1292503910.1046/j.1365-2362.2003.01216.x

[19] BarzonL, BoscaroM, PaluG (2004) Endocrine aspects of cancer gene therapy. Endocr Rev 25: 1–44.1476982610.1210/er.2002-0035

[20] WickhamTJ, MathiasP, ChereshDA, NemerowGR (1993) Integrins alpha v beta 3 and alpha v beta 5 promote adenovirus internalization but not virus attachment. Cell 73: 309–319.847744710.1016/0092-8674(93)90231-e

[21] BergelsonJM, CunninghamJA, DroguettG, Kurt-JonesEA, KrithivasA, et al (1997) Isolation of a common receptor for Coxsackie B viruses and adenoviruses 2 and 5. Science 275: 1320–1323.903686010.1126/science.275.5304.1320

[22] FechnerH, HaackA, WangH, WangX, EizemaK, et al (1999) Expression of coxsackie adenovirus receptor and alphav-integrin does not correlate with adenovector targeting in vivo indicating anatomical vector barriers. Gene Ther 6: 1520–1535.1049076110.1038/sj.gt.3301030

[23] MizuguchiH, KoizumiN, HosonoT, Ishii-WatabeA, UchidaE, et al (2002) CAR- or alphav integrin-binding ablated adenovirus vectors, but not fiber-modified vectors containing RGD peptide, do not change the systemic gene transfer properties in mice. Gene Ther 9: 769–776.1204045810.1038/sj.gt.3301701

[24] YunCO, YoonAR, YooJY, KimH, KimM, et al (2005) Coxsackie and adenovirus receptor binding ablation reduces adenovirus liver tropism and toxicity. Hum Gene Ther 16: 248–261.1576126410.1089/hum.2005.16.248

[25] ParkerAL, WaddingtonSN, NicolCG, ShayakhmetovDM, BuckleySM, et al (2006) Multiple vitamin K-dependent coagulation zymogens promote adenovirus-mediated gene delivery to hepatocytes. Blood 108: 2554–2561.1678809810.1182/blood-2006-04-008532

[26] WaddingtonSN, ParkerAL, HavengaM, NicklinSA, BuckleySM, et al (2007) Targeting of adenovirus serotype 5 (Ad5) and 5/47 pseudotyped vectors in vivo: fundamental involvement of coagulation factors and redundancy of CAR binding by Ad5. J Virol 81: 9568–9571.1755388210.1128/JVI.00663-07PMC1951445

[27] KalyuzhniyO, Di PaoloNC, SilvestryM, HofherrSE, BarryMA, et al (2008) Adenovirus serotype 5 hexon is critical for virus infection of hepatocytes in vivo. Proc Natl Acad Sci U S A 105: 5483–5488.1839120910.1073/pnas.0711757105PMC2291105

[28] WaddingtonSN, McVeyJH, BhellaD, ParkerAL, BarkerK, et al (2008) Adenovirus serotype 5 hexon mediates liver gene transfer. Cell 132: 397–409.1826707210.1016/j.cell.2008.01.016

[29] VigantF, DescampsD, JullienneB, EsselinS, ConnaultE, et al (2008) Substitution of hexon hypervariable region 5 of adenovirus serotype 5 abrogates blood factor binding and limits gene transfer to liver. Mol Ther 16: 1474–1480.1856041610.1038/mt.2008.132

[30] Groot-WassinkT, AboagyeEO, WangY, LemoineNR, ReaderAJ, et al (2004) Quantitative imaging of Na/I symporter transgene expression using positron emission tomography in the living animal. Mol Ther 9: 436–442.1500661110.1016/j.ymthe.2003.12.001

[31] Richard-FiardoP, FrankenPR, LamitA, MarsaultR, GuglielmiJ, et al (2012) Normalisation to blood activity is required for the accurate quantification of Na/I symporter ectopic expression by SPECT/CT in individual subjects. PLoS One 7: e34086.2247051710.1371/journal.pone.0034086PMC3309932

[32] FaivreJ, ClercJ, GerolamiR, HerveJ, LonguetM, et al (2004) Long-term radioiodine retention and regression of liver cancer after sodium iodide symporter gene transfer in wistar rats. Cancer Res 64: 8045–8051.1552021410.1158/0008-5472.CAN-04-0893

[33] JouretF, WalrandS, ParreiraKS, CourtoyPJ, PauwelsS, et al (2010) Single photon emission-computed tomography (SPECT) for functional investigation of the proximal tubule in conscious mice. Am J Physiol Renal Physiol 298: F454–460.1995518810.1152/ajprenal.00413.2009

[34] LoeningAM, GambhirSS (2003) AMIDE: a free software tool for multimodality medical image analysis. Mol Imaging 2: 131–137.1464905610.1162/15353500200303133

[35] MirzaM, HreinssonJ, StrandML, HovattaO, SoderO, et al (2006) Coxsackievirus and adenovirus receptor (CAR) is expressed in male germ cells and forms a complex with the differentiation factor JAM-C in mouse testis. Exp Cell Res 312: 817–830.1641000110.1016/j.yexcr.2005.11.030

[36] CanyJ, AvrilA, PichardV, AubertD, FerryN, et al (2007) A transgenic mouse with beta-Galactosidase as a fetal liver self-antigen for immunotherapy studies. J Hepatol 47: 396–403.1746278310.1016/j.jhep.2007.03.018

[37] AlbaR, BradshawAC, CoughlanL, DenbyL, McDonaldRA, et al (2010) Biodistribution and retargeting of FX-binding ablated adenovirus serotype 5 vectors. Blood 116: 2656–2664.2061081710.1182/blood-2009-12-260026PMC2974579

[38] KoskiA, RajeckiM, GuseK, KanervaA, RistimakiA, et al (2009) Systemic adenoviral gene delivery to orthotopic murine breast tumors with ablation of coagulation factors, thrombocytes and Kupffer cells. J Gene Med 11: 966–977.1967033210.1002/jgm.1373

[39] JonssonMI, LenmanAE, FrangsmyrL, NybergC, AbdullahiM, et al (2009) Coagulation factors IX and X enhance binding and infection of adenovirus types 5 and 31 in human epithelial cells. J Virol 83: 3816–3825.1915824910.1128/JVI.02562-08PMC2663266

[40] BradshawAC, ParkerAL, DuffyMR, CoughlanL, van RooijenN, et al (2010) Requirements for receptor engagement during infection by adenovirus complexed with blood coagulation factor X. PLoS Pathog. 6: e1001142.10.1371/journal.ppat.1001142PMC295138020949078

[41] RaschpergerE, ThybergJ, PetterssonS, PhilipsonL, FuxeJ, et al (2006) The coxsackie- and adenovirus receptor (CAR) is an in vivo marker for epithelial tight junctions, with a potential role in regulating permeability and tissue homeostasis. Exp Cell Res 312: 1566–1580.1654265010.1016/j.yexcr.2006.01.025

[42] HaddadD, ZanzonicoPB, CarlinS, ChenCH, ChenNG, et al (2012) A vaccinia virus encoding the human sodium iodide symporter facilitates long-term image monitoring of virotherapy and targeted radiotherapy of pancreatic cancer. J Nucl Med 53: 1933–1942.2313908810.2967/jnumed.112.105056PMC6386167

[43] BartonKN, StrickerH, BrownSL, ElshaikhM, ArefI, et al (2008) Phase I study of noninvasive imaging of adenovirus-mediated gene expression in the human prostate. Mol Ther 16: 1761–1769.1871430610.1038/mt.2008.172PMC3127288

[44] BartonKN, StrickerH, ElshaikhMA, PeggJ, ChengJ, et al (2011) Feasibility of adenovirus-mediated hNIS gene transfer and 131I radioiodine therapy as a definitive treatment for localized prostate cancer. Mol Ther 19: 1353–1359.2158720910.1038/mt.2011.89PMC3129572

[45] TajimaT, OkadaT, MaXM, RamseyW, BornsteinS, et al (1999) Restoration of adrenal steroidogenesis by adenovirus-mediated transfer of human cytochromeP450 21-hydroxylase into the adrenal gland of21-hydroxylase-deficient mice. Gene Ther 6: 1898–1903.1060238610.1038/sj.gt.3301018

[46] LymperopoulosA, RengoG, ZincarelliC, SoltysS, KochWJ (2008) Modulation of adrenal catecholamine secretion by in vivo gene transfer and manipulation of G protein-coupled receptor kinase-2 activity. Mol Ther 16: 302–307.1822354910.1038/sj.mt.6300371

[47] MatkovicU, PacentiM, TrevisanM, PaluG, BarzonL (2009) Investigation on human adrenocortical cell response to adenovirus and adenoviral vector infection. J Cell Physiol 220: 45–57.1920255510.1002/jcp.21727

[48] AlesciS, RamseyWJ, BornsteinSR, ChrousosGP, HornsbyPJ, et al (2002) Adenoviral vectors can impair adrenocortical steroidogenesis: clinical implications for natural infections and gene therapy. Proc Natl Acad Sci U S A 99: 7484–7489.1203230910.1073/pnas.062170099PMC124257

[49] WillhauckMJ, Sharif SamaniBR, KlutzK, CengicN, WolfI, et al (2008) Alpha-fetoprotein promoter-targeted sodium iodide symporter gene therapy of hepatocellular carcinoma. Gene Ther 15: 214–223.1798970510.1038/sj.gt.3303057

[50] MorleySD, ViardI, ParkerKL, MullinsJJ (1996) Adrenocortical-specific transgene expression directed by steroid hydroxylase gene promoters. Endocr Res 22: 631–639.896992210.1080/07435809609043757

